# Research Status of Mouse Models for Non-Small-Cell Lung Cancer (NSCLC) and Antitumor Therapy of Traditional Chinese Medicine (TCM) in Mouse Models

**DOI:** 10.1155/2022/6404853

**Published:** 2022-09-21

**Authors:** Hongkui Chen, Min Zheng, Wenhui Zhang, Yuan Long, Yu Xu, Man Yuan

**Affiliations:** ^1^Shanghai Lidebiotech Co. Ltd., Shanghai 201203, China; ^2^School of Pharmacy, Shanghai University of Traditional Chinese Medicine, Shanghai 201203, China; ^3^Engineering Research Center of Shanghai Colleges for TCM New Drug Discovery, Shanghai 201203, China

## Abstract

Non-small-cell lung cancer (NSCLC) is known as one of the most lethal cancers, causing more than 1 million deaths annually worldwide. Therefore, the development of novel therapeutic drugs for NSCLC has become an urgent need. Herein, various mouse models provide great convenience not only for researchers but also for the development of antitumor drug. Meanwhile, TCM, as a valuable and largely untapped resource pool for modern medicine, provides research resources for the treatment of various diseases. Until now, cell-derived xenograft (CDX) model, patient-derived xenograft (PDX) model, syngeneic model, orthotopic model, humanized mouse model (HIS), and genetically engineered mouse models (GEMMs) have been reported in TCM evaluation. This review shows the role and current status of kinds of mouse models in antitumor research and summarizes the application progress of TCM including extracts, formulas, and isolated single molecules for NSCLC therapy in various mouse models; more importantly, it provides a theoretical exploration of what kind of mouse models is ideal for TCM efficacy evaluation in future. However, there are still huge challenges and limitations in the development of mouse models specifically for the TCM research, and none of the available models are perfectly matching the characteristics of TCM, which suppress the tumor growth through various mechanisms, especially by regulating immune function. Nevertheless, with fully functional immune system existing in syngeneic model and humanized mouse model (HIS), it is still suggested that these two models are more suitable for development of TCM especially for TCM extracts or formulas. Moreover, continued efforts are needed to generate more reliable mouse models to test TCM formulas in future research.

## 1. Introduction

Lung cancer is a heterogeneous group of tumors, consisting of approximately 80 histologic, genetic, and molecularly defined subtypes, and non-small-cell lung cancer (NSCLC) accounts for approximately 85% of all these subtypes [1, 2]. WHO has classified NSCLC into 3 main types, that is, adenocarcinoma, squamous cell carcinoma, and large cell cancer, with adenocarcinoma (ADC, approximately 40–50% of cases), squamous cell carcinoma (SqCC, approximately 20–30% of cases), and large cell cancer (LCC, approximately 5–10% of cases) comprising the predominant histological subtypes of NSCLC [3, 4]. Genetic alterations, tobacco use (smoking and secondhand smoking), and environmental exposures, including air pollution, infection, and occupational exposures, have been demonstrated to be associated with the tumorigenesis of NSCLC. Based on the stage, histology, gene mutations, and patient's condition, the treatments of NSCLC usually include the surgery, radiotherapy, chemotherapy, molecularly targeted therapy, and immunotherapy [5, 6]. However, NSCLC may reoccur and metastasize when there is a high risk that patients may harbor minimal residual [7]. Traditional cytotoxic chemotherapy and radiation therapy are the most common clinical treatment strategies but are always associated with many side effects [8]. Acquired drug resistance of NSCLC cells is always related to molecularly targeted therapy, and there are most toxicities as immune-related adverse events (irAEs), which resulted from excessive immunity against normal organs in clinical trials for immunotherapy [9–12]. Thus, it is necessary to find alternative therapeutic agents for NSCLC. Consequently, with more complicated elemental structures and abundant biological activities, TCM products primarily including TCM herbals or formulas have gradually become a huge resource base upon the development of anticancer drugs due to their intrinsic advantages [13–16].

TCM products have been used for the treatment of various diseases over thousands of year in eastern Asia [17, 18]. Since there is more recognition of these diseases or disorders, an extensive number of TCM products have been identified, and many useful drugs have been developed from these products, which have played wide roles in rejuvenation, cytoprotection, anti-inflammatory, anti-infection, antioxidation, anticancer, etc. [19–25]. Currently, TCM products and their biological activities are a subject of great interest in the pharmaceutical, health food, and cosmetics industries, and numbers of scientific studies in these field are increasing rapidly [26]. And a plenty of TCM products (all of extracts, formulas, and isolated single molecules) and their analogs and metabolites may serve as the shortcut or key resources of new drug candidates for anticancer therapy. Recent studies indicated that TCM products can be used as anticancer therapy with minimum side effects and can also be used as potential MDR modulators to overcome drug resistance [27–30]. In addition, many preclinical studies on NSCLC showed positive effects of TCM products including flavonoids, diterpenoids, triterpenoids, steroids, macrodiolides, and phenolics [31–35], so there is an urgent need for NSCLC animal models suitable for development of TCM products, which will shed light on the diversity of new drug discovery for NSCLC.

During the last decades, there has been a great effort in developing preclinical animal models for NSCLC, including cell lines-derived xenografts (CDX), genetically engineered mouse models (GEMM), and patient-derived xenografts (PDX). These models have been used to accelerate our understanding of NSCLC biology and pathogenesis [36, 37]. Because preliminarily preclinical toxicity and efficacy study in animal models are an important regulatory requirement in drug development to assess the safety and activity of the test TCM products prior to clinical evaluation, in this review, we focus on the role and development of kinds of mouse models in antitumor research and summarize that the efficacy and safety of TCM products for the treatment of NSCLC in mouse models. What deserves more attention is that we should take full advantage of mouse models to reexamine the important value of TCM products in NSCLC from a new perspective. Furthermore, the lack of systemic evaluation of pharmacology and toxicology using modern methods and the not-well-identified material base of TCM extracts or formulas are the major reasons why TCM extracts or formulas are not accepted as drugs by the western world [18]; thus, we also should seek for some kinds of mouse models, which are more suitable for development of TCM extracts or formulas when compared to synthetic chemical drugs.

## 2. Classification of Animal Models

The use of preclinical models is a core component in every aspect of translational cancer research ranging from the biological understanding of the disease to the development of new treatments, so insufficiencies in preclinical animal models are key factors in the high failure rates of oncology drug discovery and development [38]. An ideal animal model should allow the development of local tumors, it should replicate all stages of cancer progression, and finally, it should permit assessment of new therapeutic strategies. Since 1970s, screening of new drugs was performed in rapidly growing mouse models. Over the last 40–50 years, xenografts developed by growing cell lines or from fresh primary or metastatic human cancer tissues subcutaneously or orthotopically in immunodeficient mice are the most commonly used *in vivo* platform in preclinical drug development [39]. The classical models for cancer drug screening include CDXs, PDXs, cell line- or primary tumor-derived homografts in syngeneic mice, orthotopic patient-derived or cell line-derived xenografts, HIS, and GEMMs [40]. The flowchart of various models establishment is shown in Figure 1.

### 2.1. Cell-Derived Xenograft (CDX) Model

CDX mouse models are developed by implanting cell lines in mice to effectively grow tumors, which emerge from xenograft transplantations and are a mosaic of human cancer cells and mouse stromal cells. Furthermore, in order for human tumors to grow in mice, the host must be immunocompromised to prevent immune rejection [37]. There are several advantages with CDXs including relatively cost-effective and good reproducibility, high tumor-take rates, short turn-around time, and maintenance of molecular characteristics from the original cell line; thus, CDXs remain invaluable for large-scale drug screening, biomarker discovery, and PK/PD analysis of new drugs, as well as exploring drug resistance mechanisms [41, 42]. Presently, over 200 cell lines for NSCLC have been reported, and many NSCLC CDX mouse models were utilized to examine the effects of TCM products [43]. However, some problems still exist in CDX models: (i) CDX models cannot reconstitute complex human cancer elements such as the molecular heterogeneity of tumor cells and the tumor microenvironment, so approximately 88% of new drugs identified by CDXs fail in clinical research [44]. (ii) CDX models lack fully functional murine immune systems [45]. Therefore, actually, till now, cell-derived xenograft (CDX) models are mainly utilized to evaluate pharmacology, efficacy, and safety profiles of TCM monomers and synthetic chemical drugs at the early stage of preclinical research.

### 2.2. Patient-Derived Xenograft (PDX) Model

Patient-derived xenografts (PDX) are based on transferring primary tumors directly from the patient into an immunodeficient mouse. To establish patient-derived xenograft (PDX) model, patient tumors must be obtained freshly from surgery, mechanically or chemically digested at once, and transplanted in immunodeficient mouse while saving a small portion as a primary stock [46]. Patient‐derived xenograft models are considered superior to cell line‐derived xenograft (CDX) models in retaining the histological characteristics of patient tumors, such as tumor heterogeneity and tumor microenvironment, at least at early passages [47]. Along with the advancement of molecular and genomic analyses, researchers have focused on more details in individual cancer genes and the tumor microenvironment; thus, PDX models are more suitable for use in experiments exploring the sensitivity of drugs, which is more similar to clinical drug responsiveness, the molecular mechanisms of tumor progression, drugs resistance, PDX biobanks, and precision medicine by which the most effective drugs can be identified in individual PDX model [48, 49]. However, there are some limitations that PDX models are expensive with a low transplantation success rate and require a long tumor-take time [50]. Currently, the number of NSCLC PDX is increasing rapidly; it will be beneficial for a better understanding of the mechanisms by which NSCLC progresses and develops resistance to certain drugs especially for targeted small molecules including TCM monomers because the major challenge in the treatment of NSCLC patients is intrinsic or acquired resistance to chemotherapy [51], but a treatment targeting may delay the development of resistance in NSCLC patients.

### 2.3. Syngeneic Model

Syngeneic murine models are to implant murine-derived cancer lines or tissues on homozygouslyinbred murine strains. Herein, murine-derived cancer lines have either been derived from chemical-induced tumors or tumors that spontaneously generate in the same strain [50]. The advantage of syngeneic models is that the transplanted cancer lines or tissues, the tumor microenvironment, and the host are from the same species. This is extremely important when considering the close interaction between tumor and host characterized by the process of metastasis. Furthermore, syngeneic models are both time- and cost-effective and reproducible [52]. The disadvantage of syngeneic models is that their model systems are short of many important characteristics of human tumors. For instance, they are generally derived from homozygously inbred mice or rats and, therefore, lack the genetic complexity of human tumors. This allows for evaluation of toxicities, including on-target/off-tumor side effects, and the immunosuppressive microenvironments [53]. Now, due to the growing worldwide enthusiasm in cancer immunotherapy, syngeneic murine models are widely used tools for studying tumor immunity and immunotherapy response because there is a fully functional murine immune system [51, 54, 55].

### 2.4. Orthotopic Model

Orthotopic models were established by directly implanting tumor cells or fresh tumor tissues into mice in the anatomical location from which they were originally derived. As a result, the use of orthotopic implantation has resulted in tumor models resembling human cancer with respect to the biology and tumor microenvironment [56, 57]. Therefore, orthotopic models allow the evaluation of tumor behavior in an organ-specific microenvironment. In addition, because the lack of metastasis and altered drug responses have been reported in commonly used subcutaneous models, the orthotopic models enhance the possibility of distant metastatic spread in a superior manner and allow to elucidate the role of certain molecular pathways by direct comparison of the metastatic properties of a given cell with their genetically engineered counterpart. The additional transfection of these cells with a reporter, like GFP, DsRed, or luciferase, allows monitoring of tumor progress by *in vivo* imaging [58, 59], which makes orthotopic models more valuable, but challenging to construct and measure the tumor size. The 90% death of non-small-cell lung cancer (NSCLC) patients is primarily due to metastases, which are poorly amenable to therapeutic intervention [60]. Many studies have shown orthotopic engraftment of human NSCLC tumors in mice for the studies of metastasis [61–65]. Therefore, the remarkable advantages of orthotopic transplantation facilitate NSCLC cancer growth in a more natural environment, which can mimic an eventual onset and spreading of metastases similar to those found in men.

### 2.5. Humanized Mouse Models (HIS)

Humanized mouse models, which are engrafted with functional human cells and tissues, including human peripheral blood mononuclear cells (PBMCs), CD34+ human hematopoietic cells, or bone marrow-liver-thymus (BLT) tissue, are widely used for the biomedical research [66]. The NSG, NCG, and NOG mouse strains are suitable for creating humanized mice because they lack T-cell subsets, B cells, and natural killer (NK) cells. For example, Hu-PBL-NSG mouse model was established by engrafting human peripheral blood mononuclear cells (PBMCs) into NOD/SCID/IL-2R*γ*−/− (NSG) mice. Then, an ALK positive cell line, H3122 (EML4-ALK variant 1), or a patient-derived tumor from EML4-ALK-rearranged (EML4-ALK variant 1) NSCLC patient was transplanted in NSG mice [48]. When engrafted with human peripheral blood mononuclear cells, tumor tissues, and immune systems, the humanized mice could recapitulate the biological responses faithfully. The humanized mouse models are now being widely used to study many human biological responses and diseases and are increasingly utilized as preclinical tools for evaluation of drugs and for identifying underlying mechanisms in the aspect of tumor immunotherapy. The recent clinical successes of immune checkpoint blockade and chimeric antigen receptor T cell therapies inspired a turning interest in cancer immunotherapy. Humanized mouse models could be a powerful animal model for testing efficacy of immunotherapeutic agents including TCM products. However, many humanized mice have a short experimental window because of the development of graft-versus-host disease (GVHD), usually within 4–8 weeks [51, 52]. Additionally, not all immune cell populations can be reconstituted in this system [67].

### 2.6. Genetically Engineered Mouse Models (GEMMs)

GEMMs of cancer represent a diverse collection of genetically modified mice, which are engineered to carry cloned oncogenes or lack tumor-suppressing genes and allow the investigation of human disease-associated genetic abnormalities *in vivo*. Such models can be divided into two forms: Germ-Line genetically engineered models, which develop cancers in an unintended (spontaneous) fashion, and conditional genetically engineered models, which provide regulated control of tumor onset utilizing tissue-specific, ligand-regulated, and/or viral-based technologies [53]. Presently, GEMMs for most of the common NSCLC driver mutations have been generated, including KRAS (Kras^LSL − G12D/+^, Kras^LSL − G12D^/ + /Tp53^mutants^, Kras^LSL − G12D/+^/Lkb1^*F/F*^, Lkb1^*F*/−^, Lkb1^*F*/+^ or Lkb1^+/−^, Kras^LSL − G12D/+^/Cdkn2a^*F/F* or −/−^, Tet-op Kras4b^G12D^/CCSP-rtTA), epidermal growth factor receptor (EGFR) (Tet-op EGFR^L858R^/CCSP-rtTA, Tet-op EGFR^L858R + T790M^/CCSP-rtTA, Tet-op EGFR^∆E746 − A750 + T790M^/CCSP-rtTA, Tet-op EGFR^T790M^/CCSP-rtTA), phosphoinositide-3-kinase catalytic alpha polypeptide (PIK3CA) (Tet-op PIK3CA^H1047R^/CCSP-rtTA) and echinoderm microtubule-associatedprotein-like 4 (EML4)–anaplastic lymphoma kinase (ALK)[ LSL-EML4-ALK^L1196M/+ or F1174L/+^, Tet-op EML4-ALK (Variant 1)/CCSP-rtTA, SPC-EML4-ALK (variant 1)] [68–70]. However, there are several disadvantages to GEMMs, including the relatively long period needed for GEMMs to develop tumor and the unpredictable nature of tumor development with regard to frequency and latency of tumorgenesis [71], which can become a drawback for preclinical evaluation of test articles including TCM.

## 3. Animal Models for Analysis and Testing of TCM Products as Chemotherapy Agents

The application of animal models has contributed remarkably to drug development. Mouse models are the most extensively used in preclinical NSCLC studies for *in vivo* analysis of tumor response to chemotherapy, which is defıned as a cytotoxic and systemic therapy that disrupts basic cellular processes such as proliferation, metastasis, maintenance, apoptosis, and angiogenesis, not just those with oncogenic drivers. Traditional Chinese Medicine products have been proved effective in cancer therapy by preventing recurrence and development of multidrug resistance with tolerable side effect and alleviated detrimental symptoms caused by standard chemotherapy. Many studies that included all NSCLC subtypes have successfully evaluated TCM products in mouse models including CDX, PDX, and orthotopic and GEMM models, and these TCM products have cytotoxic properties with many different mechanisms of action, such as the inhibition of tumor cell growth, the induction of apoptosis, DNA damage, and the inhibition of topoisomerases I and II (see Table 1).

Nevertheless, most of these TCM products, usually acting as isolated single molecules, which are similar to synthetic chemical drugs [18], may also increase the risk of TCM molecules induced adverse effects. Simultaneously, long history has proved TCM herbals or formulas to be of benefit over the risk of induced adverse effects, but it is noticed that TCM herbals or formulas mainly play a supporting role in the main treatment.

## 4. Animal Models for Analysis and Testing of TCM Products as Targeted Therapy Agents

There is now a better understanding of the role of driver mutations in NSCLC and how to target these mutations in treatment of NSCLC, for example, epidermal growth factor receptor (EGFR) mutation, ROS1-rearranged, BRAF^V600E^ mutation, KRAS mutation, and anaplastic lymphoma kinase (ALK) fusion oncogene [98]. Although currently applicable to only a minority of patients with NSCLC, this development has resulted in prominent successes that have led to approved molecularly specific, biomarker-defined indications for targeted therapies. However, most of the available anticancer agents are designed to target specific driver mutations by altering the activity of involved transporters and genes. As cancer cells demonstrate complex cellular machinery, the regeneration of cancer tissues and drug resistance towards the therapy has been the main barrier in cancer treatment [99]. A plenty of TCM products, as a valuable and huge resource pool, exhibited multitargeted characteristics of antioxidant, antimitotic, anti-inflammatory, antibiotic, and anticancer activity. Therefore, this fact encourages the researchers to explore the multitargeted use of TCM products especially for monomers to overcome the shortcomings and seek alternative and safer treatment strategies. Many preclinical studies included the fact that TCM monomers were used in NSCLC treatment for multitargeted approach (see Table 2).

## 5. Animal Models for Analysis and Testing of TCM Products as Immunotherapy Agents

Lung cancer has traditionally been considered as a “nonimmunogenic” malignancy. However, the recent advancement about using immunotherapy to treat NSCLC has been driven by remarkable results from clinical studies evaluating antibodies to programmed death receptor 1 (PD-1) and programmed death ligand 1 (PD-L1). Immunotherapy is generally well tolerated and has demonstrated a survival benefit in patients with advanced NSCLC. On the one hand, many immunotherapeutic agents, including monoclonal antibodies and small molecules, have shown significant antitumor activity in NSCLC humanized mouse models *in vivo*. Therefore, without doubt, humanized mouse models could be an extremely important animal model for pursuing novel immunotherapy treatment strategies in advanced NSCLC. The evidence is that many of TCM products including Polyphenols (e.g., Curcumin, Resveratrol), Cardiotonic Steroids (e.g., Digoxin and Bufalin), Terpenoids (e.g., Paclitaxel, Artemisinin, and Triptolide), Polysaccharides (e.g., Lentinan), Saponins, and Capsaicin have potential immunomodulatory effects [113], so increasing the focus has been driven toward finding novel potential modulators of tumor immunotherapy from TCM products. Maybe these TCM products combined with immune checkpoint inhibitor can be further studied in humanized mouse models and exert their advantages in immunotherapy for NSCLC, with synergistic effects and reduced toxicity [114]. On the other hand, syngeneic mouse models used for preclinical studies including intact immune responses also can provide a closer correlation with human cancer, especially for TCM products, like herbal medicines and monomeric compound, having great potential for targeting immune modulators [115–118]. In addition, TCM formulas have made great breakthroughs in the treatment of NSCLC by regulating the body to suppress tumors on the whole [8]. Meanwhile, a number of studies have shown that TCM formulas suppress the proliferation of cancer cells through various mechanisms especially by regulating immune function. The efficacy and mechanism of TCM formulas in the therapy of NSCLS in syngeneic mouse models are summarized as follows (see Table 3).

## 6. Outlook and Challenges

Humans have been using TCM products to treat diseases for thousands of years [122]. TCM can regulate the proliferation, adhesion, apoptosis, and tumor migration and inhibit tumor angiogenesis and change immune system. Actually, the mechanism of action of many TCM products is still unclear, but the therapeutic effects of TCM products on various diseases and immune regulation have been proved [123]. Although many TCM products have been reported on antitumor and immune modulatory effects, the research and application of TCM are still limited. The current researches are mainly focused on the TCM isolated single molecules, following the evaluation system of chemical drugs. However, TCM is usually used in the form of formulas rather than individual purified molecules. The composition of many TCM formulas, usually administered orally, is extraordinarily complex and metabolized to more complex metabolites in the body. Therefore, it is challenging to evaluate the efficacy of TCM by *in vitro* experiments, including cell based assay.

The *in vivo* models can mimic the metabolism and distribution of drugs in the body; therefore, they are more suitable for evaluating the antitumor effect of TCM. However, there are limited reports about the application of TCM formulas, compared to the chemical drug or antibodies, in animal models, and most of the reported models are CDXs and syngeneic mouse models. As an important tool in antitumor research, mouse models have always been the gold standard to evaluate the antitumor activity of drugs [124]. In view of the fact that TCM formulas usually act on multiple targets and signal pathways and may have the function of regulating immunity, animal models with complete immune system function are more suitable for the efficacy study of TCM formulations. Both syngeneic mouse models and humanized models have fully functional immune system and are powerful tools to evaluate the anticancer efficacy of TCM objectively. Considering the cost and difficulty of modeling, it is suggested that syngeneic mouse models could be utilized for testing the antitumor activities of TCM formulas in the early research, and humanized models could be used in further research.

The high incidence of NSCLC and the high rate of recurrence and metastasis in postoperative patients result in the urgent demand for more kinds of effective drugs. At present, targeted drugs and immune drugs have provided more treatment options and helped prolong the lives for cancer patients. But there are still unsolved problems in toxicity, effectiveness, and drug resistance of antitumor drugs. As a massive resource pool, TCM products provide powerful resources for finding new drugs for NSCLC patients. However, due to the lack of the support of large-scale preclinical and clinical research based on the concept of evidence-based medicine, TCM can only be regarded as an adjuvant therapy in the standard treatment of NSCLC. Until now, there is no animal model developed specifically for the TCM research, and none of the available models are perfectly matching the mechanism or characters of TCM, especially TCM formulas. Although syngeneic mouse and humanized models can be used in TCM studies, the establishment of more suitable models would be a valuable and promising field of research. It is believed that, with the development of research tool and deeper exploration of TCM products, more efficacy studies on mouse tumor models will be carried out, facilitating the development of antitumor drugs.

## Figures and Tables

**Figure 1:** The flowchart of various models' establishment.

**Table 1:** List of TCM products as chemotherapy agents reported anticancer effects in NSCLC models.

TCM products	Origin	NSCLC models	Underlying mechanisms
Taxanes including paclitaxel and docetaxel	Paclitaxel derived from the bark of the Pacific yew, docetaxel is a semi-synthetic taxane derived from extracts of the European yew tree *Taxus baccata*	A549 (Adenocarcinoma), H1299 (Lack expression of p53 protein)	Tubulin inhibitor, which interferes with the normal function of cellular microtubule growth by binding to the *β*-subunits of the tubulin and locking the microtubules preventing further cell division [33, 72, 73].
Vincaleucoblastine including vindesine and vinorelbine	Vindesine is a vinca-alkaloid derived from *vinblastine*, vinorelbine is a semisynthetic vinca-alkaloid	Lu-65 (Lung large cell carcinoma) and PC-12 (Adenocarcinoma); the EGFR-wild-type A549 and the EGFR-mutated (exon 21 L858R/exon 20 T790M) H1975 [74]	Tubulin inhibitor, the mechanism of action is the inhibition of tubulin polymerization into microtubules.
Evodiamine	A novel alkaloid, isolated from the fruit of *Tetradium*	H1975 (Adenocarcinoma)	NF-kB inhibitor, by downregulation of MUC1-C [75–77].
Honokiol	Purified from the magnolia tree	PC‐9/AR (EGFR _19del), PC‐9/3M [(EGFR-19del, T790M, C797S (cis)], A549,H1299, acquired resistance to cetuximab in NSCLC patient-derived xenograft (PDX) model	By overcoming Osim acquired resistance [78], being associated with induction of apoptotic cell death and inhibition of class I HDACs proteins and HDAC activity [79, 80].
Sinomenine	Purified from the roots of the plant *Sinomenium acutum*	HCC827 (Adenocarcinoma), H1975	By reducing HK2-mediated glycolysis [81].
Formononetin	Originated mainly from red clovers and the Chinese herb *Astragalus membranaceus*	HCC827, H3255 (Adenocarcinoma), H1975, A549, H1299 [82]	By inducing cell cycle arrest, apoptosis, antiangiogenesis, and metastasis [83].
Quercetin	As the active compound from Yang-Yin-Qing-Fei-Tang (YYQFT), which is a well-known traditional Chinese medicine	A549, HCC827	Through induction of apoptosis or autophagy, enhancement of chemosensitivity, and modulation of cancer stemness [84, 85].
Isoharringtonine (IHT)	As an alkaloid extracted from the leaves of *Cephalotaxus koreana Nakai*.	A549	Inhibition of the growth of tumor spheroids, induced apoptotic cell death via the Intrinsic pathway [86].
MTE (M. Tenacissima extract)	Extracted from *Marsdenia tenacissima* (Roxb.) *Wight & Arn*	H1975	Inhibiting ABCG2 activity, by elevating production of NO, in a PKA-dependent manner [87, 88].
Chlorella sorokiniana	Extracted from *Chlorella*	CL1-5 (Adenocarcinoma)	Downregulation of Bcl-2, XIAP and survival [89].
Yuanhuadine (YD; purity >98.5%)	Isolated from a CHCl3-soluble fraction of the flowers of *Daphne genkwa*	Acquired Gefitinib-resistantpatient-derived xenograft (PDX) model	By complete suppression of the AXL activation [90].
Feiji Recipe	As a classical herbal recipe	2LL-EGFP-Ido orthotopic xenografts	By reducing IDO expression [91].
Cyclopamine tartrate (CycT), an improved analogue of Cyclopamine	Cyclopamine produced by *Veratrum californicum* being a rich source of steroidal alkaloids and growing in high mountain meadows	Orthotopically implanted H1299-luc NSCLC tumor xenografts	Inhibitor of the hedgehog (hh) signaling pathway [92–94].
Baicalein	Derived from the root of *Scutellaria*	A549 orthotopic xenografts	By inhibition of Id1 expression [89].
Yi-Fei-Jie-Du-Tang (YFJDT)	As a traditional Chinese medicine formula	A549	Through upregulating FAT4, promoting autophagy [16].
Theabrownin	Derived from the green tea	H1299 (p53-deficient) and A549 (p53-wild type)	By the activation of MAPK/JNK signaling pathway [95].
Ze-Qi-Tang formula	As a traditional Chinese medicine	LLC orthotopic mouse model	By inducing apoptosis via STAT3/S100A9/Bcl-2/caspase-3 signaling [96].
BL02 formula	Consists of two herbs: *Gentiana rhodantha Franch. Ex Hemsl* and *Gerbera anandria*	HCC827 and A549 orthotopic xenografts	Inhibition of Rap1/cdc42 signaling [97].

**Table 2:** List of TCM products as targeted therapy agents reported anticancer effects in NSCLC models.

Natural products	Origin	NSCLC models	Underlying mechanisms
Tanshinone IIA	Isolated from the rhizome of the Chinese herb *Salvia miltiorrhiza Bunge* (danshen)	HCC827/gefitinib _resistant, A549 [100]	VEGFR inhibitor, via regulation of VEGFR/Akt pathway [101], suppression of EGFR signaling [102, 103] and downregulation of the expression levels of Bcl‐2, Caspase‐3, p‐Akt, and p‐PI3K proteins [104]
Parthenolide	Originated from the medicinal plant feverfew (*Tanacetum parthenium*)	H1975, H460, A549	By targeting EGFR through downregulation of ERK and AKT expression [105]
Hydroxygenkwanin (HGK)	One of the active flavonoids extracted from the flower buds of *Daphne genkwa Sieb.et Zucc*.	H1975	By inducing the proteasome-mediated degradation of EGFR, thus inhibiting EGFR-downstream signaling and inducing apoptosis [106]
Deguelin	Derived from leguminous plants	HCC827, H1975, A549 and H3255	By inhibiting EGFR signaling and promoting GSK3*β*/FBW7-mediated Mcl-1 destabilization. [107, 108]
Baicalein	Derived from the root of *Scutellaria baicalensis*	H1299	Binding to MAP4K3 and degradation of MAP4K3 [109]
Diaporine A (D261)	Derived from the culture broth of endophytic fungus *Diaporthe* sp. *3lp-10*	NCI–H460	By regulating miR-99a/mTOR signaling [110]
Thevebioside	An active ingredient from the seed of *Thevetia peruviana* (pers) *K. Schum* (TPKS).	A549	By inhibiting SRC mediated IGF-1R–PI3K-AKT signaling [111].
Compounds of tanshinone (CTN)	Extracted from *Salvia miltiorrhiza Bunge* roots	GLC-82 (Adenocarcinoma)	By inducing apoptosis through the mitochondrial pathway of apoptosis and PTEN-mediated inhibition of PI3K/Akt pathway [112]
Toona sinensis leaf extract	Extracted from *Toona sinensis* leaves	H441 (Adenocarcinoma), H520 (squamous cell carcinoma) and H661 (Large cell cancer)	Downregulation of cyclin D1 and CDK4 by increasing the expression of cyclin-dependent inhibitor p27 [89]

**Table 3:** List of TCM formulas as targeted therapy agents reported anticancer effects in NSCLC models.

Formulas	Origin	NSCLC models	Underlying mechanisms
Bu-Fei decoction	Consisting of six herbal Chinese medicines including *Codonopsis pilosula*, *Schisandra chinensis*, *Rehmannia glutinosa*, *Astragalus*, *Aster* and *Cortex Mori.*	H1975, A549	Partially via IL-10 and PD-L1 regulation [119].
Yangyinwenyang (YYWY)	Consisting of *Paris polyphylla* var, *yunnanensis*, *Gynostemma pentaphyllum*, *Ophiopogon intermedius D. Don,* and *Trigonella foenum-graecum L*	The Lewis lung cancer cells in C57BL/6 female mice	Through facilitating the mature DCs to activate the proliferation and differentiation of T cells [120].
Hedyotis diffusa willd	*Hedyotis diffusa Willd* extract powder	The Lewis lung cancer cells in C57BL/6 female mice	May activate immunity, achieve anti-inflammatory, antiproliferative, and antimigration therapeutic effects by regulating multiple pathways.
Yu-ping-Feng (YPF)	Composed of *Astragali Radix* (huangqi), *Atractylodis Macrocephalae Rhizoma* (Baizhu), and *Saposhnikoviae Radix* (Fangfeng)	The Lewis lung cancer cells in C57BL/6 female mice	Downregulated the expression of TGF-*β*, indoleamine 2, 3-dioxygenase, and IL-10 in tumor microenvironment and had a NK cell-dependent inhibitory effect on Lewis lung cancer [121].
